# lncRNA FOXD2-AS1 Promotes the Retinoblastoma Cell Viability and Migration by Sponging miR-31

This article has been retracted.

**DOI:** 10.1155/2022/7723425

**Published:** 2022-06-23

**Authors:** Yan Liang, Hong Wang, Ruiying Song, Xiuyan Yin

**Affiliations:** Department of Ophthalmology, The Affiliated Yantai Yuhuangding Hospital of Qingdao University, Yantai, 264000 Shandong Province, China

## Abstract

**Background:**

The purpose of this study was to explore the functions of FOXD2-AS1 and miR-31 in retinoblastoma. *Material and Methods*. An RT-qPCR assay was applied to calculate the mRNA levels of FOXD2-AS1, miR-31, and PAX9. A dual-luciferase reporter gene assay was employed to verify the connection between FOXD2-AS1, miR-31, and PAX9 expression.

**Results:**

FOXD2-AS1 was upregulated, and miR-31 was lowly expressed in retinoblastoma. Low expression of FOXD2-AS1 promoted cell proliferation and migration, and upregulation of FOXD2-AS1 inhibited proliferative and migratory abilities. lncRNA FOXD2-AS1 directly bound to miR-31 and regulated miR-31 expression in SO-RB50 cells. Cell proliferation and migration were inhibited by the miR-31 mimic. miR-31 mediated PAX9 expression via directly binding to PAX9 mRNA. A miR-31 inhibitor partially reversed the effect of FOXD2-AS1 knockdown on the proliferation and migration in SO-RB50 cells. FOXD2-AS1 knockdown reduced PAX9 expression in SO-RB50 cells. PAX9 had negative connection with miR-31, and it had positive relationship with FOXD2-AS1.

**Conclusion:**

lncRNA FOXD2-AS1 inhibited cell proliferation and migration via the miRNA-31/PAX9 axis in retinoblastoma.

## 1. Introduction

Retinoblastoma (RB) is the most frequent intraocular malignancy in childhood caused by the mutation of the RB1 gene [1]. Approximately 8000 cases of retinoblastoma are diagnosed worldwide each year, and the mortality rate in developing countries is about 70% [2, 3]. Retinoblastoma is usually observed with choroidal infiltration of the eye pathologically. The tumor begins to spread from the retina to the sclera and laminar posterior optic nerve and even metastasize to the central nervous system of advanced retinoblastoma [4]. The overall survival rate of patients after metastasis will decrease significantly. Thus, it is urgent to explore the molecular mechanism of retinoblastoma treatment to enhance clinical treatment effect.

Long noncoding RNAs (lncRNAs), longer than 200-nucleotide RNAs, acted as key regulators in eukaryotic transduction [5, 6]. Increasing evidence indicates that lncRNAs have broad prospects as a novel biomarker and therapeutic target for cancer, including retinoblastoma [7]. For instance, lncRNA SNHG16 enhanced cell proliferation and colony formation and inhibited cell apoptosis in retinoblastoma [8]. Upregulation of FOXD2-AS1 was associated with tumor progression and metastasis in papillary thyroid cancer [9]. Long noncoding RNA FOXD2-AS1 functioned as a competitive endogenous RNA by sponging miRNAs in several cancers, including hepatocellular carcinoma, thyroid cancer, esophageal squamous cell carcinoma, and glioma [10–13]. lncRNAs acted as miRNAs' competing endogenous RNA (ceRNA) or “RNA sponges” and were related to the progression of multiple tumors including cell growth, metastasis, and cell apoptosis [14].

MicroRNAs (miRNAs) are short noncoding RNA molecules that contain 19-25 nucleotides [15, 16]. miRNAs can mediate gene expression by binding to the 3′-untranslated region (3′-UTR) complementary sequence of the target mRNAs, eventually leading to mRNA degradation or reduced translation [17]. As tumor-suppressive miRNAs, miR-31 suppressed cell viability, metastasis, and cell cycle in renal cell carcinoma [18]. Downregulation of miR-31 suppressed cell proliferation and invasion via Wnt/*β*-catenin signaling in osteosarcoma [19]. Moreover, miR-31 was lowly expressed and played great roles in gastric cancer, nasopharyngeal carcinoma, and oral cancer, while it was overexpressed in colorectal cancer [20–23]. In this study, we found that FOXD2-AS1 inhibited cell proliferation and migration via the miRNA-31/PAX9 axis in retinoblastoma.

## 2. Material and Methods

### 2.1. Patients and Specimens

We collected 38 freshly frozen retinoblastoma tissue specimens from patients who received surgery at Affiliated Yantai Yuhuangding Hospital of Qingdao University between January 2015 and June 2019. The mean age of the retinoblastoma patients was 3.6 years ranging from 2 months to 11 years. And 12 normal retina samples were obtained from patients with globe rupture. All tumor tissues were examined by two independent histopathologists and graded according to guideline issues by the 7th edition of the American Joint Committee on Cancer.

### 2.2. Cell Culture

Tree human retinoblastoma cells (SO-RB50, Y79, and Weri-RB1) and a normal retinal pigmented epithelial cell line ARPE-19 were obtained from ATCC. All cells were cultured in DMEM containing 10% fetal bovine serum at 37°C in a humidified incubator supplied with 5% CO_2_.

### 2.3. Cell Transfection

The sh-FOXD2-AS1, miR-613 mimic, and miR-613 inhibitor together with their control sequences were all purchased from GenePharma (Shanghai, China). FOXD2-AS1 was inserted into a pcDNA3.1 vector (Sangon, Shanghai, China) to construct a FOXD2-AS1 overexpression vector. SO-RB50 cells were cultured overnight to achieve 70–80% confluence prior to transfection. Thereafter, the transfection was performed in SO-RB50 cells using Lipofectamine 2000 (Invitrogen).

### 2.4. qRT-PCR

Ribozol was used to extract total RNAs from RB tissues and cells. In brief, the reverse transcription was performed to synthesize the first-strand cDNA chain using AMV Reverse Transcriptase XL (Clontech, USA). To detect the expression of FOXD2-AS1, qPCR was carried out using SYBR Green Master Mix (Bio-Rad, USA) on an ABI 7500 System. All experiments were performed 3 times, and the data were processed using the 2^−ΔΔCT^ method. qRT-PCR primers were as follows: FOXD2-AS1 forward: 5′-TGGACCTAGCTGCAGCTCCA-3′ and reverse: 5′-AGTTGAAGGTGCACACACTG-3′; PAX9 forward: 5′-ACCACATTTACTCATATCCCAGTCCCA-3 and reverse: 5′-GGCTCCCTTCTCCAATCCATTCA-3′; GAPDH forward: 5′-TATGATGATATCAAGAGGGTAGT-3′ and reverse: 5′-TGTATCCAAACTCATTGTCATAC-3′; miR-31 forward: 5′-ACGCGGCAAGATGCTGGCA-3′ and reverse: 5′-CAGTGCTGGGTCCGAGTGA-3′; and U6 forward: 5′-CTCGCTTCGGCAGCACA-3′ and reverse: 5′-AACGCTTCACGAATTTGCGT-3′.

### 2.5. Proliferation Assay

For the detection of cell proliferation, the CCK-8 assay (Beyotime, Jiangsu, China) was performed. SO-RB50 cells were seeded into 96-well plates and incubated for 1, 2, 3, or 4 days. Subsequently, each well was added with the CCK-8 reagent followed by incubation of the cells for an additional 4 h. The absorbance at 450 nm was evaluated on a microplate reader.

### 2.6. Scratch Test

After 48 hours of transfection, cells were cultured at 5 × 10^5^ cells per well in 6-well plates. After complete adherence to the wall, the cells were scratched with a cell scraper in the middle of each well and then cultured for 24 hours. Photographs were taken at 0 h and 24 h after scratching, and the scratch distance was computed with Image-Pro Plus 6.0. The experiments were repeated three times at least.

### 2.7. Transwell Assay

Cell migration was assessed by using a transwell chamber in a 24-well plate. In brief, the upper chamber was seeded with 200 *μ*l cells suspended with medium without FBS, whereas the bottom chamber was filled with complete medium with 20% FBS. After incubation for 24 h, cells still on the upper chamber were removed using cotton swabs. Meanwhile, the migrated cells were fixed using paraformaldehyde for 15 min and then stained using crystal violet. The migrated cells were counted in five randomly selected fields under light microscopy (Olympus, Tokyo, Japan).

### 2.8. Dual-Luciferase Reporter Assay

Starbase was used to predict FOXD2-AS1 binding to miR-31. TargetScan predicted the potential targets of miR-31, and finally, the putative complementary sequence of which was identified in the 3′-UTR of PAX9 mRNA. SO-RB50 cells were cotransfected with the miR-31 mimic and wild-type or mutated PAX9 or FOXD2-AS1. The Lipofectamine 2000 reagent (Invitrogen) was employed to carry out the transfection. After transfection for 48 h, the dual-luciferase reporter assay system was utilized to calculate the luciferase activity. The firefly luciferase activity was evaluated and normalized by Renilla luciferase activity.

### 2.9. Statistical Analysis

Data were expressed as mean ± standard deviation (SD). The SPSS 20.0 software package (SPSS, Chicago, IL, USA) was employed to carry out the statistical analysis. The differences between two groups were analyzed using the Student *t*-test and Fisher's exact tests. One-way analysis of variance (ANOVA) and Bonferroni post hoc tests were used to compare three or more groups. Pearson correlation between FOXD2-AS1, miR-31, and PAX9 was assessed in RB tissues.

## 3. Results

### 3.1. Upregulation of FOXD2-AS1 in Retinoblastoma

To detect the functions of FOXD2-AS1 in retinoblastoma, the expression of FOXD2-AS1 was calculated using RT-qPCR. As expected, FOXD2-AS1 was upregulated in 38 retinoblastoma tissues versus 12 normal retina samples (*P* < 0.05) (Figure 1(a)). Similarly, the RT-qPCR assay demonstrated that FOXD2-AS1 was also overexpressed in RB cells SO-RB50, Y79, and WERI-RB1 versus normal cell ARPE-19 (*P* < 0.05) (Figure 1(b)). We also explored evidence for a correlation between FOXD2-AS1 expression and clinicopathological status in glioma patients. The results indicated that significant correlations were detected between FOXD2-AS1 expression and certain clinicopathological features, including lymph node metastasis and IIRC stage (*P* < 0.05) (Table 1).

### 3.2. FOXD2-AS1 Promotes the Proliferative Ability in SO-RB50 and Y79 Cells

To detect the biological effects of FOXD2-AS1 in SO-RB50 and Y79 cells, sh-FOXD2-AS1 and pEX-FOXD2-AS1 were constructed. The transfection efficiency of FOXD2-AS1 knockdown (*P* < 0.05) or overexpressed FOXD2-AS1 (*P* < 0.05) was calculated using RT-qPCR (Figures 2(a) and 2(c)). The CCK-8 assay was conducted to measure the cell proliferation after transfecting sh-FOXD2-AS1 or pEX-FOXD2-AS1 in SO-RB50 and Y79 cells. As we discovered, silencing of FOXD2-AS1 reduced cell proliferation in SO-RB50 and Y79 cells (*P* < 0.05) (Figure 2(b)). In contrast, cell proliferation was enhanced after transfecting pEX-FOXD2-AS1 in SO-RB50 cells compared with control groups (*P* < 0.05) (Figure 2(d)).

### 3.3. FOXD2-AS1 Enhances Cell Migratory Ability in SO-RB50 and Y79 Cells

In addition, the transwell assay was employed to evaluate the cell migration after transfecting sh-FOXD2-AS1 or pEX-FOXD2-AS1 in SO-RB50 and Y79 cells. Similarly, cell migration was reduced when FOXD2-AS1 is knocked down (*P* < 0.05). On the contrary, upregulation of FOXD2-AS1 enhanced cell migratory ability in SO-RB50 and Y79 cells (*P* < 0.05) (Figure 3(a)). In addition, the scratch test was used to further measure the migratory ability in SO-RB50 and Y79 cells. The results indicated that in comparison with the sh-NC group, the migration of cells in the sh-FOXD2-AS1 group was distinctly lessened. On the contrary, overexpression of FOXD2-AS1 promoted cell migratory ability in SO-RB50 and Y79 cells (Figure 3(b)).

### 3.4. FOXD2-AS1 Targets miR-31 in Retinoblastoma

Starbase was utilized to predict the potential target miRNAs of FOXD2-AS1, and we selected miR-31 as the research object. To test whether FOXD2-AS1 binds to miR-31, the potential binding sequences were mutated from UCUUGC to UGAACC, and both the wild-type or the mutant FOXD2-AS1 was inserted in the psiCHECK-2 plasmid (Promega, Madison, WI, USA) (Figure 4(a)). The luciferase assay revealed that luciferase activity was reduced when the miR-31 mimic and wild-type FOXD2-AS1 were cotransfected in SO-RB50 cells (*P* < 0.05). Meanwhile, the luciferase activity has no alteration after cotransfection with the miR-31 mimic and mutant FOXD2-AS1 (Figure 4(b)). In addition, miR-31 mRNA level was calculated after up- or downregulation of FOXD2-AS1 in SO-RB50 cells. Not unfortunately, miR-31 was reduced by overexpression of FOXD2-AS1 (*P* < 0.05) (Figure 4(c)). In addition, the expression of miR-31 has a negative connection with FOXD2-AS1 in retinoblastoma tissues (*P* < 0.05) (Figure 4(d)).

### 3.5. miR-31 Inhibits Cell Viability and Migration in SO-RB50 Cells

To explore the roles of miR-31 in retinoblastoma, the expression of miR-31 was measured using RT-qPCR. Contrary to the level of FOXD2-AS1, miR-31 was lowly expressed in retinoblastoma tissues in comparison with normal retina samples (*P* < 0.05) (Figure 5(a)). Also, miR-31 was downregulated in RB cells SO-RB50, Y79, and WERI-RB1 versus normal cell ARPE-19 (*P* < 0.05) (Figure 5(b)). To investigate the functions of miR-31, the miR-31 mimic was used to overexpress miR-31 in SO-RB50 cells, and the transfection efficiency was calculated using RT-qPCR (*P* < 0.05) (Figure 5(c)). CCK-8 results indicated that the miR-31 mimic impaired SO-RB50 cell proliferation (*P* < 0.05) (Figure 5(d)). Moreover, cell migration was suppressed by the miR-31 mimic through the transwell assay (*P* < 0.05) (Figure 5(e)).

### 3.6. miR-31 Targets PAX9 in Retinoblastoma

TargetScan was utilized to predict the potential target genes of miR-31, and we selected PAX9 as a target of miR-31. To explore the functions of miR-31 in mediating retinoblastoma cells, the predicted binding sequences on PAX9 were mutated (Figure 6(a)). After that, both the wild-type and the mutant PAX9 together the with miR-31 mimic were cotransfected in SO-RB50 cells. The luciferase reporter assay indicated that the miR-31 mimic reduced the luciferase activity of wild-type PAX9 (*P* < 0.05), and the miR-31 mimic has no effect on the mutant PAX9 (*P* < 0.05) (Figure 6(b)). PAX9 expression was calculated after overexpression of miR-31 in SO-RB50 cells, and we discovered that PAX9 expression was reduced by the miR-31 mimic (*P* < 0.05) (Figure 6(c)). Pearson correlation was used to evaluate the relationship between PAX9 and miR-31 in SO-RB50 cells, and we found that it had a negative correlation between them (Figure 6(d)).

### 3.7. FOXD2-AS1 Regulates Cell Proliferation and Migration via the miR-31/PAX9 Axis

To investigate the molecular mechanism of FOXD2-AS1 in retinoblastoma, the miR-31 inhibitor was transfected in FOXD2-AS1-silenced SO-RB50 cells (*P* < 0.05) (Figure 7(a)). The function experiment revealed that the miR-31 inhibitor partially reversed the proliferation (*P* < 0.05) and migration (*P* < 0.05) of FOXD2-AS1 in SO-RB50 cells (Figures 7(b) and 7(c)). Moreover, PAX9 expression was calculated when transfecting sh-FOXD2-AS1, and we found that it was decreased in SO-RB50 cells (*P* < 0.05) (Figure 7(d)). In addition, there is connection between PAX9 and FOXD2-AS1 in retinoblastoma tissues, and we found that it had a positive relationship between PAX9 and FOXD2-AS1 (*P* < 0.05) (Figure 7(e)).

## 4. Discussion

Retinoblastoma occurs in the retina and is a rare tumor of childhood with an incidence of 1/15,000-20,000 [1]. Specifically, retinoblastoma has the highest prevalence in Asia and Africa, with a mortality rates of about 40-70% [24]. Therefore, a new biomarker is urgently needed to treat retinoblastoma.

lncRNAs are noncoding RNAs larger than 200 nucleotides [25]. Accumulating evidence indicated that lncRNAs played great functions in retinoblastoma. For instance, lncRNA SNHG16 enhanced metastasis by LASP1 in retinoblastoma [26]. FOXD2-AS1 knockdown inhibited cell viability and motility and promoted their apoptosis [27]. Similarly, FOXD2-AS1 acted as an oncogene in hepatocellular carcinoma by accelerating cell cycle, cell colony formation, and cell proliferation [28]. In this study, we discovered that FOXD2-AS1 was overexpressed in retinoblastoma cells and tissues. Consistent with the above studies, we found that interference of FOXD2-AS1 promoted retinoblastoma cell proliferation and migration, and cell proliferation and migration were inhibited by overexpressing FOXD2-AS1.

lncRNAs often played roles in promoting or inhibiting tumor development via sponging miRNA. For example, lncRNA LOC554202 enhanced acquired gefitinib resistance through sponging miR-31 in NSCLC [29]. UCA1 promoted cell proliferation and multidrug resistance of retinoblastoma cells through sponging miR-513a [30]. In our study, FOXD2-AS1 was used as a ceRNA to adsorb miR-31. The expression of miR-31 was reduced after overexpression of FOXD2-AS1, and it was increased by FOXD2-AS1 knockdown. MicroRNAs (miRNAs) are small noncoding RNAs by binding to target genes to mediate gene expression [31, 32]. miR-31 inhibited cell proliferation, migration, and invasion via targeting PIK3C2A [33]. Moreover, miR-31 regulated chemosensitivity through preventing the nuclear location of PARP1 in HCC [34]. Our findings were consistent with the previous studies; miR-31 was lowly expressed in retinoblastoma tissues and cells. Since miR-31 was lowly expressed in retinoblastoma cells, we used the miR-31 mimic to overexpress miR-31 in SO-RB50 cells. Moreover, the miR-31 mimic inhibited cell proliferation and migration in SO-RB50 cells. Thus, we proposed that FOXD2-AS1 enhanced retinoblastoma cell proliferation and invasion via regulating miR-31. In addition, the results of this current study indicated that PAX9 expression was regulated by miR-31, and PAX9 was determined to be a target gene of miR-31. Except that, silencing of FOXD2-AS1 could inhibit the expression of PAX9, indicating that FOXD2-AS1 suppresses miR-31 expression, thereby promoting PAX9 expression.

## 5. Conclusion

FOXD2-AS1 was used as a ceRNA to adsorb miR-31 for suppressing its expression, thereby promoting PAX9 expression. Our study provided a new insight into how FOXD2-AS1 can be an effective target for retinoblastoma diagnosis. However, we only studied the functions of FOXD2-AS1 on retinoblastoma in vitro, so in vivo experiments are needed, which is the limitation of this article.

## Figures and Tables

**Figure 1:** Upregulation of FOXD2-AS1 in retinoblastoma tissues and cells: (a) FOXD2-AS1 was upregulated in retinoblastoma tissues compared with normal retina samples; (b) FOXD2-AS1 was also overexpressed in RB cells.

**Figure 2:** FOXD2-AS1 promoted cell proliferative ability in SO-RB50 and Y79 cells: (a) the transfection efficiency of FOXD2-AS1 knockdown in SO-RB50 and Y79 cells using RT-qPCR; (b) silencing of FOXD2-AS1 reduced cell proliferation in SO-RB50 and Y79 cells; (c) overexpressed FOXD2-AS1 was calculated using RT-qPCR; (d) cell proliferation was enhanced after pEX-FOXD2-AS1 transfection in SO-RB50 and Y79 cells.

**Figure 3:** FOXD2-AS1 enhanced cell migratory ability in SO-RB50 and Y79 cells: (a) transwell assay was used to measure cell migration in SO-RB50 and Y79 cells; (b) scratch test was applied to calculate cell migratory ability in SO-RB50 and Y79 cells.

**Figure 4:** FOXD2-AS1 targets miR-31 in retinoblastoma: (a) miR-31 was predicted to target miRNA of FOXD2-AS1; (b) luciferase activity was reduced when the miR-31 mimic and wild-type FOXD2-AS1 were cotransfected in SO-RB50 cells; (c) miR-31 mRNA level was calculated after FOXD2-AS1 up- or downregulation in SO-RB50 cells; (d) the expression of miR-31 has a negative connection with FOXD2-AS1 in retinoblastoma tissues.

**Figure 5:** miR-31 inhibited cell viability and migration in SO-RB50 cells: (a) miR-31 was lowly expressed in retinoblastoma tissues in comparison with normal retina samples; (b) miR-31 was downregulated in RB cells; (c) the transfection efficiency of transfecting the miR-31 mimic in SO-RB50 cells using RT-qPCR; (d) miR-31 mimic impaired SO-RB50 cell proliferation; (e) cell migration was suppressed by the miR-31 mimic through the transwell assay.

**Figure 6:** miR-31 targets PAX9 in retinoblastoma: (a) TargetScan predicted that PAX9 was a target of miR-31; (b) luciferase assay was performed to verify miR-31 binding to PAX9; (c) PAX9 expression was reduced by the miR-31 mimic; (d) it had a negative correlation between PAX9 and miR-31 in SO-RB50 cells.

**Figure 7:** FOXD2-AS1 regulates cell proliferation and migration via the miR-31/PAX9 axis: (a) miR-31 inhibitor was transfected in FOXD2-AS1-silenced SO-RB50 cells; (b) miR-31 inhibitor partially reversed the proliferation of FOXD2-AS1; (c) miR-31 inhibitors can partially reverse the effect of FOXD2-AS1 on motility in SO-RB50 cells; (d) PAX9 expression was decreased in SO-RB50 cells; (e) it had a positive relationship between PAX9 and FOXD2-AS1.

**Table 1:** The expression of FOXD2-AS1 and clinicopathological features in 38 paired retinoblastoma.

Clinicopathological features	Cases (*n* = 38)	FOXD2-AS1 expression		*P* value^∗^
		15 high (%)	23 low (%)	
Gender				0.944
Male	18	7 (38.9)	11 (61.1)	
Female	20	8 (40.0)	12 (60.0)	
Lymph node metastasis				0.017^∗^
No	14	9 (64.3)	5 (35.7)	
Yes	24	6 (25.0)	18 (75.0)	
IIRC stage				0.036^∗^
Group A-B	15	9 (60.0)	6 (40.0)	
Group C-E	23	6 (26.1)	17 (73.9)	

^∗^Statistically significant difference (*P* < 0.05).

## Data Availability

Data to support the findings of this study is available on reasonable request from the corresponding author.
